# Selected Enzyme Inhibitory Effects of* Euphorbia characias* Extracts

**DOI:** 10.1155/2018/1219367

**Published:** 2018-05-29

**Authors:** Antonella Fais, Benedetta Era, Amalia Di Petrillo, Sonia Floris, Dario Piano, Paola Montoro, Carlo Ignazio Giovanni Tuberoso, Rosaria Medda, Francesca Pintus

**Affiliations:** ^1^Department of Sciences of Life and Environment, University of Cagliari, Cittadella Universitaria, 09042 Monserrato, Italy; ^2^Department of Pharmacy, University of Salerno, 84084 Fisciano, Italy

## Abstract

Extracts of aerial part of* Euphorbia characias* were examined to check potential inhibitors for three selected enzymes involved in several metabolic disorders. Water and ethanol extracts from leaves and flowers showed* in vitro *inhibitory activity toward *α*-amylase, *α*-glucosidase, and xanthine oxidase. IC_50_ values were calculated for all the extracts and the ethanolic extracts were found to exert the best effect. In particular, for the *α*-glucosidase activity, the extracts resulted to be 100-fold more active than the standard inhibitor. The inhibition mode was investigated by Lineweaver-Burk plot analysis.* E. characias* extracts display different inhibition behaviors toward the three enzymes acting as uncompetitive, noncompetitive, and mixed-type inhibitors. Moreover, ethanolic extracts* of E. characias* showed no cytotoxic activity and exhibited antioxidant capacity in a cellular model. The LC-DAD metabolic profile was also performed and it showed that leaves and flowers extracts contain high levels of quercetin derivatives. The results suggest that* E. characias* could be a promising source of natural inhibitors of the enzymes involved in carbohydrate uptake disorders and oxidative stress.

## 1. Introduction

Oxidative stress and Reactive Oxygen Species (ROS) are involved in the development of various human diseases. Many cellular enzymes as well as nonenzymatic processes are potential sources of free radicals, which lead to oxidative stress. Accordingly, ROS could originate from different physiological and pathological pathways, where, in the latest case, they may induce several levels of cellular stresses and apoptosis. In this respect, an example is represented by the enzyme xanthine oxidase (EC 1.2.3.2), which may provide a significant contribution in generating ROS by the oxidation reaction of hypoxanthine and xanthine to uric acid, yielding superoxide radicals O2^•−^. Overproduction or reduced excretion of uric acid leads to abnormal amounts of uric acid in the body, causing hyperuricemia and gout. This metabolic disorder is associated with the crystallization and deposition of uric acid in joints and surrounding tissue, causing inflammation, gouty arthritis, and uric acid nephrolithiasis [1]. Xanthine oxidase inhibitors are indicated for treatment of hyperuricemia and gout. They can alleviate the symptoms of inflammatory-associated diseases by the reduction of uric acid synthesis and they have a key role in decreasing oxidative stress [2].

Another contribution in ROS production, under either physiological or pathological conditions, derives from disease related to the primary metabolism such as diabetes. Increasing hyperglycemia is believed to be connected with the production of free radicals and ROS, leading to oxidative tissue damage and diabetic complications [3]. Diabetes mellitus is a progressive metabolic disorder of glucose metabolism. Type 1 diabetes results from inadequate synthesis of insulin by pancreatic *β*-cells, while type 2 diabetes is characterized primarily by insulin resistance or *β*-cell dysfunction [4]. The early stage of diabetes mellitus type 2 is associated with postprandial hyperglycemia due to impaired after meal acute insulin secretion. Therefore, a therapeutic approach to treat diabetes is to decrease postprandial hyperglycemia [4]. This can be achieved by the inhibition of carbohydrate hydrolyzing enzymes like *α*-amylase and *α*-glucosidase that break down starch and disaccharides to glucose, thereby moderating the postprandial blood glucose elevation [5]. *α*-Amylase (EC 3.2.1.1) catalyzes the endohydrolysis of *α*-D-1,4-glycosidic bonds in starch, producing maltose and various oligosaccharides. *α*-Glucosidase (EC 3.2.1.3) catalyzes the hydrolysis of terminal 1,4-linked *α*-D-glucose residues from nonreducing ends of isomaltose oligosaccharides, yielding free D-glucose.

Plants have become a prolific source of structurally diverse bioactive molecules and the bioactivity of some of them is linked to their antioxidant activity. The effects of plant materials could result from isolated substances but typically derive from the synergy of different bioactive compounds present in the plant. Medicinal plants have been evaluated for their inhibitory and antioxidant activities in treatment of gout [6–9]. Several inhibitors of *α*-amylase and *α*-glucosidase have been isolated from medicinal plants to serve as an alternative drug with increased potency and lesser adverse effects than existing synthetic drugs [10–12].

Phytochemical and pharmacological studies have reported a wide spectrum of medicinal properties of the genus* Euphorbia*, revealing an important biological potential [13]. Euphorbiaceae are a large plant family comprising more than 300 genera and 8,000 species. Among the Euphorbiaceae, the species* Euphorbia characias* is a typical shrub commonly occurring in vast areas of the Mediterranean basin. The plant latex has been object of extended research and its screening has revealed the presence of antioxidants and acetylcholinesterase inhibitors [14], a natural rubber [15], and various enzymes [16–18], some of these interacting in a common metabolism [19]. Besides the latex, recently the attention has been paid also to other parts of the plant [20, 21]. In particular, aerial parts of* E. characias* were examined for their antioxidant, antimicrobial, anti-HIV, and cholinesterase inhibitory activities [22]. Moreover, leaves, stems, and flowers exhibited antimelanogenic effect in cell-free and cellular systems [23].

The objective of this research was to extend the characterization of this plant as potential source of bioactive molecules which could be useful for pharmaceutical applications. Leaves and flowers extracts were investigated for their inhibitory activities toward *α*-amylase, *α*-glucosidase, and xanthine oxidase as well as for their oxygen radical absorbance capacity and antioxidant effect in cells.

## 2. Materials and Methods

### 2.1. Reagents

All chemicals were obtained as pure commercial products and used without further purification.

Acetonitrile, 3-O-caffeoylquinic acid (chlorogenic acid), 2′,7′-dichlorofluorescein diacetate (DCFH-DA), 3-(4,5-dimethylthiazol-2-yl)-2,5-diphenyltetrazolium bromide (MTT), fluorescein sodium salt (FL), 4-hydroxypyrazolo(3,4-d)pyrimidine (allopurinol), 6-hydroxy-2,5,7,8-tetramethylchromane-2-carboxylic acid (Trolox), phosphoric acid 85% w/v, quercetin, xanthine, and xanthine oxidase from bovine milk were purchased from Sigma-Aldrich (Milan, Italy). Standards of kaempferol-3-*O*-glucoside, quercetin-3-*O*-glucoside, ellagic acid, and acacetin were purchased from Extrasynthese (Genay Cedex, France). HPLC grade water (MΩ•cm) was prepared by using a Millipore (Bedford, MA, USA) Milli-Q purification system. Acetonitrile, water, and formic acids (all of LC-MS grade) were purchased from Merck (Darmstadt, Germany).

### 2.2. Spectrophotometric and Fluorometric Analyses

Spectrophotometric determinations were obtained with an Ultrospec 2100 spectrophotometer (Biochrom Ltd., Cambridge, England) using a 1 cm in length path cells and with a plate reader FLUOstar OPTIMA (BMG Labtech, Offenburg, Germany). The latter instrument was used also for fluorescence measurements.

### 2.3. Plant Materials

*E. characias* was previously identified [22] and a voucher specimen has been deposited (number 1216/16, Herbarium CAG). Leaves and flowers of* E. characias* were collected from February to June in southern Sardinia (Dolianova, CA; GPS coordinates were 39°24′ 19.0^″^ N and 9°12′ 57.6^″^ E) and were immediately frozen at −80°C and then lyophilized. The lyophilized plant materials were extracted in water or ethanol as previously reported [22]. Before use, 1 mg of dried powders was dissolved in water or 10% ethanol (1 mL) for water and ethanol extracts, respectively.

### 2.4. Enzymatic Inhibition

The results of all the assays described below were expressed as percentage of the blank control. Concentrations of extracts resulting in 50% inhibition of enzyme activity (IC_50_) were determined by interpolation of dose-response curves. The inhibition mode was determined performing assays at different concentrations of substrate and extracts. Kinetics data were analyzed using the Lineweaver-Burk plot.

### 2.5. Assay for *α*-Amylase Inhibitory Activity

The inhibition of *α*-amylase activity by* E. characias* extracts was determined by using 2-chloro-p-nitrophenyl-*α*-D-maltotrioside (CNPG3) as artificial substrate. A reaction mix containing 60 *μ*L of 50 mM sodium phosphate buffer at pH 7.0, 20 *μ*L of NaCl (1 M), and 40 *μ*L of *α*-amylase from porcine pancreas (1 mg/mL) was used. The solution was mixed in microplate multiwells and incubated in absence or presence of plant extracts at 37°C for 10 min. Similarly, the standard inhibitor acarbose was used as positive control. After incubation, 80 *μ*L of a 2.5 mM CNPG3 solution was added and the amount of 2-chloro-nitrophenol released by the enzymatic hydrolysis was monitored at 405 nm.

### 2.6. Assay for *α*-Glucosidase Inhibitory Activity

The effect of the plant extracts on *α*-glucosidase activity was determined by measuring the yellow-colored p-nitrophenol released from the chromogenic substrate p-nitrophenyl-*α*-D-glucopyranoside (pNPG). The enzyme solution contained 40 *μ*L *α*-glucosidase from* Saccharomyces cerevisiae* (0.125 U/mL) and 120 *μ*L of 0.1 M phosphate buffer, pH 6.9. 20 *μ*L of test samples at various concentrations was mixed with the enzyme solution in microplate wells and subsequently incubated for 15 min at 37°C. A volume of 20 *μ*L of substrate solution (5 mM pNPG) was added and incubated for an additional 15 min. The reaction was stopped by adding 50 *μ*L of 0.2 M sodium carbonate solution. Absorbance was then measured with a microplate reader at 405 nm. The systems without either plant extracts or acarbose were used as control and positive control, respectively.

### 2.7. Assay for Xanthine Oxidase Inhibitory Activity

The inhibitory effect of* E. characias* extracts on xanthine oxidase activity was determined spectrophotometrically by monitoring the formation of uric acid at 295 nm. The reaction mixture contained 879 *μ*L of 100 mM phosphate buffer, pH 7.5, 50 *μ*L of an aqueous solution of xanthine oxidase from bovine milk (0.5 U/mL, Sigma Chemical Co.), and 10 *μ*L of extract sample solution or control sample solution (ethanol or water). After mixing, 61 *μ*L of xanthine solution 0.82 mM was added and the enzyme activity was determined at 295 nm for 3 min at 25°C. Allopurinol was used as positive control.

### 2.8. Oxygen Radical Absorbance Capacity (ORAC) Assay

The ORAC assay was carried out as previously described [24]. Trolox and fluorescein (FL) were used as a standard and as a fluorescent probe, respectively. Free radicals were produced by 2,2′-azobis(2-methylpropionamidine) (AAPH) to oxidize FL. Different dilutions of Trolox (25, 12.5, 6.25, 3.13, and 1.56 *μ*M) and appropriate dilutions of the tested sample were prepared in phosphate buffer 10 mM at pH 7.4. A volume of 25 *μ*L of Trolox or sample solution was pipetted into a well of a 96-well black microplate, and then FL (150 *μ*L, 10 nM) was added. The reaction mixture was incubated at 37°C for 30 min. Afterwards, at the excitation wavelength of 485 nm, emission was measured every 90 s at 520 nm. After 3 cycles, AAPH (25 *μ*L, 240 mM) was added quickly, and then the measurement was resumed and continued up to 90 min. The background signal was determined using the first 3 cycles.

### 2.9. Cell Culture and Intracellular ROS Levels

Murine melanoma B16F10 cells (CRL-6475) were purchased from the American Type Culture Collection (ATCC, Manassas, VA, USA). The cells were cultured in Dulbecco's Modified Eagle's Medium (DMEM) containing 10% fetal bovine serum (FBS, Gibco, NY, USA) and 1% penicillin/streptomycin at 37°C in a humidified atmosphere with 5% CO_2_. Cell viability was detected by the colorimetric 3-(4,5-dimethylthiazol-2-yl)-2,5-diphenyltetrazolium bromide (MTT) assay as previously described [25]. After 24 h incubation with extracts at different concentrations (0–150 *μ*g/mL), cells were labelled with MTT solution for 3 h at 37°C. The resulting violet formazan precipitates were dissolved in isopropanol and the absorbance of each well was determined at 590 nm using a microplate reader with a 630 nm reference.

The cellular ROS levels were determined with the 2′,7′-dichlorofluorescein diacetate (DCFH-DA) method [26]. B16F10 melanoma cells were treated with various concentrations of extracts (0–150 *μ*g/mL) for 24 h. Then, the cells were incubated with 10 mM H_2_O_2_ at 37°C for 30 min. After incubation, DCFH-DA (10 *μ*M) was added to the wells, and the cells were cultured for 30 min. Following this treatment, the cells were washed with phosphate-buffered saline solution and harvested. The fluorescence intensity of DCF was measured at excitation wavelength of 504 nm and emission wavelength of 524 nm by using a fluorescent plate reader.

### 2.10. LC-ESI-Orbitrap MS, LC-ESI-Orbitrap MS/MS, and LC-DAD

Qualitative investigation of the extracts was performed by LC-ESI-Orbitrap MS and LC-ESI-Orbitrap MS/MS as reported in previous work [22]. The electrospray ionization (ESI) source of a Thermo Scientific LTQ-Orbitrap XL (Thermo Scientific, Germany) mass spectrometer was tuned in negative ion mode with a standard solution of kaempferol-3-*O*-glucoside as previously reported [22]. In the FT experiment, resolution of the Orbitrap mass analyzer was set at 30000 and the mass spectrometric spectra were acquired by full range acquisition covering *m*/*z* 250–1200 in LC-MS. The data recorded were processed with Xcalibur 2.0 software (Thermo Fisher Scientific). LC-ESI-LIT-Orbitrap MS was performed using a Finnigan Surveyor HPLC (Thermo Fisher, San Jose, CA, USA) equipped with a Waters (Milford, MA, USA) XSelect CSH C18 3.5 *μ*m column (150 mm × 2.1 mm i.d.) and coupled to an hybrid Linear Ion Trap (IT) Orbitrap mass spectrometer (Thermo Scientific). Linear gradient elution with a mobile phase comprising water acidified with 0.1% formic acid (solvent A) and acetonitrile acidified with 0.1% formic acid (solvent B) as described by Pisano et al. [22] was used. The mass spectrometer was operated in negative ion mode. ESI source parameters were as follows: capillary voltage, −12 V; tube lens voltage, −121.47; capillary temperature, 280°C; sheath and auxiliary gas flow (N2), 30 and 5; sweep gas, 0, and spray voltage, 5 V. MS spectra were acquired by full range acquisition covering *m*/*z* 150–1600. LC-ESI-(LIT) MS/MS data were obtained by applying a Data Dependent Scan experiment by directing to fragmentation the highest two peaks obtained in LC-ESI-Orbitrap-MS trace. Each parent ion was submitted to fragmentation with energy of 30% to produce an MS/MS spectrum in the specific MS range relative to its mass. 10 *μ*L was injected in the system, prepared by dissolving 1 mg of dried extract in 10 mL of a mixture of water in acetonitrile.

Quantitative analysis of phenolic compounds was carried out using an HPLC-DAD method [22]. Chromatograms and spectra were elaborated with a ChromQuest V. 2.51 data system (ThermoQuest, Rodano, Milan, Italy). Flavonols were detected and quantified at 360 nm, and all the other compounds at 280 nm. The calibration curves for each compound were calculated by regression analysis by plotting the peak area obtained after standards injection (3 replicates at each concentration) against the known standard concentrations. The stock solutions were diluted with methanol in order to obtain work solutions and the correlation values were 0.9994–0.9999.* E. characias* flower extract was dissolved in methanol and injected in the LC-DAD system with the same condition of the LC-MS analysis.

## 3. Results and Discussion

### 3.1. Extract Inhibitory Activity

The effects of* E. characias* extracts on the selected enzyme activities are reported in Table 1. The results show that almost all extracts have an inhibitory activity against *α*-amylase, *α*-glucosidase, and xanthine oxidase even if they show different efficiency. Overall, ethanol extracts exert a higher effect if compared with the corresponding water extracts. We have therefore focused our attention on ethanol extracts in order to investigate the mode of inhibition of these enzymes.

The *α*-amylase inhibitory activity of* E. characias* samples reveals that the ethanol extracts (IC_50_ = 25.41 and 29.39 *μ*g/mL for leaves and flowers, resp.) were about 3.5-fold more active than the water extracts (IC_50_ = 74.02 and 109.12 *μ*g/mL for leaves and flowers, resp.). Considering that plant extracts are mixtures of numerous compounds, the real concentration of active compounds is lower than the IC_50_ value. Thus, it is not surprising that the IC_50_ values of extracts are higher than the positive control acarbose, as a single molecule (IC_50_ = 8.04 *μ*g/mL).

This provides pharmacological basis for the presence of compounds that may be effective in treatment of disorders in carbohydrate uptake.

The mode of inhibition of the ethanolic leaves extract on *α*-amylase revealed that this extract acts as a noncompetitive inhibitor. In fact, by increasing the concentration of extract, a family of straight lines with different slope, all intersecting on the abscissa, was found (Figure 1(a)). This kinetic analysis indicates that the extract can bind not only with the free enzyme but also with the enzyme-substrate complex. The equilibrium constants for binding with the free enzyme, *K*_*i*_ = 7.22 *μ*g/mL, and with the enzyme-substrate complex, *K*_*i*_′ = 7.14 *μ*g/mL, were obtained from the slope or the 1/*V*_max⁡_ values (*y*-intercepts) versus inhibitor concentration, respectively.

Lineweaver-Burk plot for flower extract showed that the extract displayed a near noncompetitive inhibition of the enzyme activity with *K*_*i*_ and *K*_*i*_′ values of 1.29 and 8.72 *μ*g/mL, respectively (Figure 1(a)).

*α*-Glucosidase activity is strongly inhibited by* E. characias* extracts (Table 1) with IC_50_ values ranging from 0.8 to 1.4 *μ*g/mL. Surprisingly, values for ethanol extracts are about 100-fold lower than the positive control, acarbose (IC_50_ = 90 *μ*g/mL). These results make* E. characias* leaves and flowers extremely interesting for further investigation in order to find novel and efficient *α*-glucosidase inhibitors.

The mode of inhibition of the ethanolic leaves extract on *α*-glucosidase displayed a noncompetitive inhibition of the enzyme (Figure 1(b)). *K*_*i*_ and *K*_*i*_′ were 0.019 and 0.017 *μ*g/mL, respectively.

The kinetic analysis of flowers extract instead produces a family of parallel lines for increasing extract concentration, indicating that this extract acts as an uncompetitive inhibitor (Figure 1(b)). The equilibrium constant for binding with the enzyme-substrate complex (*K*_*i*_′) was calculated from the replot of the intercepts (1/*V*_max⁡_) versus the inhibitor concentration, resulting in a value of 0.26 *μ*g/mL.

Ethanol extracts from leaves and flowers of* E. characias* also inhibit xanthine oxidase, although with a less efficiency if compared with the activity on the other two enzymes, showing IC_50_ of 68.9 *μ*g/mL and 85.5 *μ*g/mL, respectively. No effect was detected with aqueous extracts. The kinetic behavior of xanthine oxidase at different concentrations of xanthine and ethanol extracts is shown in Figure 1(c). Both extracts act as mixed-type inhibitor and the values of *K*_*i*_ and *K*_*i*_′ were 23.04 and 337.4 *μ*g/mL, respectively, for leaves extract and 24.5 and 812.3 *μ*g/mL, respectively, for flowers extract.

The results are comparable and are sometimes better than those of other plant extracts [6, 7, 10–12], suggesting that leaves and flowers from* E. characias* may be promising sources of enzyme inhibitors.

### 3.2. Extract Antioxidant Capacity, Cell Viability, and Intracellular ROS Levels

Since oxidative stress is considered as a key factor in the pathogenesis of some diseases such as diabetic complications, antioxidant capacity of extracts has been analyzed.

In our previous study, we have evaluated the antioxidant capacity of aerial parts of* E. characias* extracts by using FRAP, ABTS^•+^, and DPPH^•^ assays, and ethanolic extracts of leaves have shown the higher antioxidant activity [22]. In the present work, we have extended the analysis using ORAC assay, which utilizes a biologically relevant radical source. The results have confirmed the better antioxidant proprieties of leaves' ethanolic extract (data not shown).

Moreover, we also examined whether* E. characias* extracts inhibited H_2_O_2_-induced ROS generation in a cellular system.

First, the effects of leaves and flowers ethanol extracts from* E. characias* on cell viability were evaluated in B16F10 melanoma cells in order to determine the cytotoxicity of these extracts. The results indicate that both extracts are not considered to be cytotoxic in B16F10 melanoma cells (Figure 2).

To confirm the antioxidant capacity of* E. characias* extracts in a cellular model, we evaluated ROS levels in cells treated with leaves or flowers extracts before and after oxidative stress. The study was conducted using DCFH-DA, which easily diffuses through the cell membrane and is hydrolyzed by the endogenous esterases to DCFH. Rapid increases in DCF indicate the oxidation of DCFH by intracellular ROS such as H_2_O_2_. As shown in Figure 3, H_2_O_2_ incubation significantly increased ROS formation in B16F10 cells, but treatment with leaves or flowers extract decreased H_2_O_2_-induced ROS production in a dose-response manner. Thus, these results confirm the antioxidant assays and suggest that* E. characias* extracts may reduce the formation of ROS in cells.

### 3.3. Qualitative-Quantitative Determination of Phenolic Compounds in* E. characias* Extracts by (HR) LC-ESI-Orbitrap-MS, (HR) LC-ESI-Orbitrap-MS/MS, and LC-DAD Analysis

Extracts obtained from* E. characias* flowers and leaves were qualitatively analyzed by LC-ESI-Orbitrap-MS and (HR) LC-ESI-Orbitrap-MS/MS in negative ion mode. The LC-DAD method allowed quantifying the polyphenolic compounds identified by LC-MS.  Table 2 reports the detected compounds identified by High-Resolution Mass Spectrometric Data, listed according to their retention times, the quantitative amount, the chemical formula derived by accurate mass measurement, MS/MS results, and the references used for identification. Qualitative-quantitative analysis of* E. characias* flowers has been reported for the first time.

The negative LC-MS profile highlighted the presence of a large group of compounds corresponding to the deprotonated molecular ions of different phenolic derivatives, mainly flavonoids (Figure 4). Individual components were identified by comparison of their* m/z* values in the Total Ion Current (TIC) profile with those of the selected compounds described in literature (Table 2).

LC-ESI-Orbitrap-MS/MS experiments were run in order to submit the major ions to fragmentation experiments using the source and trap parameters previously selected by ESI/MS and ESI-MS/MS direct introduction experiments. By comparing experimental MS/MS spectra with fragmentation patterns reported in literature for the same analytes or with the fragmentation patterns and spectra reported in a public repository of mass spectral data, Mass Bank [27] compounds** 1**–**16** were identified, with the exception of compounds** 1**,** 2**,** 3**, and** 4** (unknown compounds).

Compounds** 6**,** 8**,** 9**,** 10**, and** 14** were identified as derivatives of quercetin by the diagnostic [M-H]^−^ ions shown in HR ESI-MS analysis. Their fragmentation profiles, obtained in LC-ESI-Orbitrap-MS/MS in Product Ion Scan and negative ion mode when compared with literature data, resulted in compounds previously reported in* E. characias* leaves [21, 22]. Quercetin-3-(2-*O*-acetyl)-arabinoside (**14**) and quercetin-3-*O*-rhamnoside (**10**) were the most abundant compounds in both flowers and leaves (47.89 ± 1.30 and 36.62 ± 0.94 g/L and 41.22 ± 1.84 and 29.80 ± 1.61, resp.). Compound** 5** was tentatively identified by the diagnostic [M-H]^−^ ion shown in HR ESI-MS analysis and by the fragmentation profile obtained in LC-ESI-Orbitrap-MS/MS working by Product Ion Scan in negative ion mode, compared with Mass Bank data. It was proposed as another quercetin derivative and probably an isomer of quercetin-3-*O*-glucoside. Myricetin-deoxyhexose, which was putatively described in leaves, was not confirmed in flowers based on fragmentation. Compound** 16** was identified by the [M-H]^−^ ion shown in HR ESI-MS and the characteristic fragmentation as quercetin previously reported in* E. characias* leaves [21]. Compound** 7** was tentatively assigned to be ellagic acid, never reported for* E. characias*. This compound was confirmed by HPLC-DAD with pure standard comparison and its amount in flower extracts was 0.57 ± 0.01 g/L. Interestingly, some ellagitannins derivatives were detected in* E. characias* leaves' ethanolic extract but were found to be absent in flowers' extracts.

The identity of compound** 11 **was hypothesized from the MS/MS data obtained by working with a LC-ESI-Orbitrap-MS/MS in Product Ion Scan and negative ion mode. A single compound was tentatively identified by Mass Bank, as dicaffeoylquinic acid, which previously was putatively described in leaves [22].

Compounds** 12** and** 13** found in the flowers were tentatively identified as derivatives of kaempferol by their [M-H]^−^ ions shown in HR ESI-MS analysis and their fragmentation profile obtained in LC-ESI-Orbitrap-MS/MS [28]. Their amount is quite low; however, they represent an interesting finding, as no kaempferol derivatives were detected in* E. characias* leaves previously [22]. Compound** 15** was tentatively identified by its [M-H]^−^ ions shown in HR ESI-MS analysis and by the fragmentation profile obtained in LC-ESI-Orbitrap-MS/MS, as derivative of acacetin, and specifically acacetin glucuronide. The amount of this compound was found to be higher in flowers' extract than in leaves' one (0.89 ± 0.07 and 0.44 ± 0.01, resp.).

## 4. Conclusions

Some enzymes play an essential role in producing ROS and they result as the main enhancers of the ROS-induced stress. Dysfunction of these enzymes results in several diseases and their therapy involves the use of specific inhibitors of their activity.

In the present study, investigation of* E. characias* extracts revealed a significant inhibitory capacity toward key enzymes (*α*-amylase and *α*-glucosidase) linked to metabolic diseases such as type 2 diabetes and gout with the prooxidant enzyme xanthine oxidase. Both these enzymes play an essential role in promoting the physiopathology of their related diseases so that any new molecule with proved inhibitory activity against them represents a new therapeutic potential. Both extracts, ethanolic or aqueous, from either leaves or flowers, showed inhibitory activity. Among them, the ethanolic extracts showed a much more pronounced activity with respect to the aqueous ones. In particular, a strong *α*-glucosidase inhibitory effect, quantified as ~100 times higher than the standard inhibitor acarbose, was found to be associated with the ethanolic extracts. Moreover, these extracts have also been shown to exert antioxidant capacity by reducing the formation of ROS in cells. The LC-DAD metabolic profile revealed that ethanolic extracts contain high levels of quercetin derivatives, which could be responsible for both the antioxidant activity and the inhibitory properties of the extracts.

Further experiments are ongoing in order to isolate the single active components responsible for the observed enzyme inhibitory activities.

## Figures and Tables

**Figure 1:** Inhibition of *α*-amylase, *α*-glycosidase, and xanthine oxidase enzymatic activities by* E. characias* ethanol extracts. Reaction conditions are reported in Materials and Methods. (a) Lineweaver-Burk plot for inhibition of *α*-amylase at different extract concentrations (*μ*g/mL). Leaves: 0 (●), 0.015 (○), 0.025 (▲), and 0.03 (∆); flowers: 0 (●), 0.025 (○), 0.03 (▲), and 0.05 (∆). (b) Lineweaver-Burk plot for inhibition of *α*-glucosidase at different extract concentrations (*μ*g/mL): 0 (●), 0.5 (○), 0.75 (▲), and 1.0 (∆). (c) Lineweaver-Burk plot for inhibition of xanthine oxidase at different extract concentrations (*μ*g/mL): 0 (●), 20 (○), 40 (▲), and 60 (∆).

**Figure 2:** Effect of* E. characias* ethanol extracts on B16F10 melanoma cell viability. After 24 h incubation with leaves (○) or flowers (●), cell viability was determined by MTT assay. Data are expressed as mean ± SD from three independent experiments.

**Figure 3:** Effect of* E. characias* ethanol extracts (25, 50, 100, and 150 *μ*g/mL) on B16F10 melanoma cells treated (T) with hydrogen peroxide (10 mM) and compared with nontreated cells (NT). White and grey bars represent flowers and leaves extracts, respectively.

**Figure 4:** (HR) LC-ESI-Orbitrap-MS analysis of* E. characias *flowers. Chromatographic conditions are described in the text. List of compounds is reported in Table 2.

**Table 1:** Inhibitory effects (IC_50_) of *E. characias* extracts on enzymatic activities. Acarbose and allopurinol are reported as standard inhibitors. All data represent the mean ± SD of three independent experiments.

Part of plant	Extract	IC_50_ (*μ*g/mL)		
		*α*-Amylase	*α*-Glucosidase	Xanthine oxidase
Leaves	Aqueous	74.02 ± 3.06	1.4 ± 0.11	>200
	Ethanolic	25.41 ± 1.42	0.8 ± 0.03	68.9 ± 6.6
Flowers	Aqueous	109.12 ± 10.36	1.1 ± 0.07	>200
	Ethanolic	29.39 ± 1.41	0.9 ± 0.04	85.5 ± 6.4
Acarbose		8.04 ± 0.65	90 ± 7.3	
Allopurinol				0.012 ± 0.0017

**Table 2:** Identification of polyphenolic compounds in *E. characias* extracts using HPLC-ESI-FT-MSMS in negative ion mode and quantification by LC-DAD.

	Putative identification	RT (min)	g/L (mean ± SD)		MW	[M-H]^−^	Molecular formula	MSMS	References
			Flowers	Leaves					
**1**	Unknown	17.31	NQ	ND	-	353.0870	C_16_H_17_O_9_	191.05	

**2**	Unknown	18.43	NQ	ND	-	799.0616	C_16_H_31_O_36_	781.04 479.04 300.99	

**3**	Unknown	19.58	NQ	NQ	-	951.0724	C_23_H_35_O_40_	933.06	

**4**	Unknown	25.05	NQ	ND	-	951.0732	C_23_H_35_O_40_	933.06 613.04	

**5**	Quercetin-glucoside (Isomer)^a^	26.77	3.95 ± 0.04	ND	464.0954	463.0873	C_21_H_19_O_12_	301.07	[22]

**6**	Quercetin-3-*O*-glucoside^*∗*^	27.12	5.87 ± 0.10	2.06 ± 0.17	464.0954	463.0873	C_21_H_19_O_12_	301.07	[21]

**7**	Ellagic acid^*∗*^	27.52	0.57 ± 0.01	ND	302.0120	301.0200	C_14_H_6_O_8_	257.10	[27]

**8**	Quercetin-3-*O*-xyloside^a^	28.70	6.09 ± 0.02	1.89 ± 0.05	434.0849	433.0771	C_20_H_17_O_11_	301.25	[21]

**9**	Quercetin-3-*O*-arabinoside^a^	29.52	21.70 ± 0.68	11.37 ± 0.22	434.0849	433.0771	C_20_H_17_O_11_	353.10 191.02	[21]

**10**	Quercetin-3-*O*-rhamnoside^a^	30.49	36.62 ± 0.94	29.80 ± 1.61	448.1005	447.0924	C_21_H_19_O_11_	329.02	[21]

**11**	di-*O*-Caffeoylquinic acid^b^	30.67	0.03 ± 0.00	0.02 ± 0.00	516.0962	515.0800	C_17_H_23_O_18_	329.02	[22]

**12**	Kaempferol-3-*O*-arabinoside^c^	33.16	0.02 ± 0.00	ND	418.0900	417.0815	C_20_H_17_O_10_	285.04	[27]

**13**	Kaempferol-3-*O*-rhamnoside^c^	34.39	0.04 ± 0.01	ND	431.0973	431.0866	C_20_H_19_O_12_	285.03	[27]

**14**	Quercetin-3-(2-*O*-acetyl)-arabinoside^a^	35.00	47.89 ± 1.30	41.22 ± 1.84	476.0954	475.0877	C_22_H_19_O_12_	301.026	[21]

**15**	Acacetin glucuronide^d^	39.14	0.89 ± 0.07	0.44 ± 0.01	460.1005	459.0980	C_22_H_19_O_11_	283.03	[22]

**16**	Quercetin^*∗*^	41.06	0.31 ± 0.04	0.02 ± 0.00	302.0236	301.0347	C_15_H_10_O_7_	178.99 151.00	[21]

“*∗*”: quantified using corresponding authentic standard; “a”: quantified as equivalent of quercetin-3-*O*-glucoside; “b”: quantified as equivalent of chlorogenic acid; “c”: quantified as equivalent of kaempferol-3-*O*-glucoside; “d”: quantified as equivalent of acacetin; ND: not detected (<LOD); NQ: detected but not quantified.

## Data Availability

The data used to support the findings of this study are available from the corresponding author upon request.

## References

[1] Richette P., Bardin T. (2010). Gout. *The Lancet*.

[2] Gliozzi M., Malara N., Muscoli S., Mollace V. (2016). The treatment of hyperuricemia. *International Journal of Cardiology*.

[3] West I. C. (2000). Radicals and oxidative stress in diabetes. *Diabetic Medicine*.

[4] Chakrabarti R., Rajagopalan R. (2002). Diabetes and insulin resistance associated disorders: disease and the therapy. *Current Science*.

[5] Oboh G., Ademosun A. O. (2011). Shaddock peels (Citrus maxima) phenolic extracts inhibit *α*-amylase, *α*-glucosidase and angiotensin I-converting enzyme activities: A nutraceutical approach to diabetes management. *Diabetes & Metabolic Syndrome: Clinical Research & Reviews*.

[6] Ling X., Bochu W. (2014). A review of phytotherapy of gout: perspective of new pharmacological treatments. *Die Pharmazie*.

[7] Orban-Gyapai O., Lajter I., Hohmann J., Jakab G., Vasas A. (2015). Xanthine oxidase inhibitory activity of extracts prepared from polygonaceae species. *Phytotherapy Research*.

[8] Kostić D. A., Dimitrijević D. S., Stojanović G. S., Palić I. R., Dordević A. S., Ickovski J. D. (2015). Xanthine oxidase: Isolation, assays of activity, and inhibition. *Journal of Chemistry*.

[9] Ansari K. A., Akram M., Asif H. M. (2011). Xanthine oxidase inhibition by some medicinal plants. *International Journal of Applied Biology and Pharmaceutical Biotechnology*.

[10] Nair S. S., Kavrekar V., Mishra A. (2013). In vitrostudies on alpha amylase and alpha glucosidase inhibitory activities of selected plant extracts. *European Journal of Experimental Biology*.

[11] Kazeem M. I., Adamson J. O., Ogunwande I. A. (2013). Modes of inhibition of *α*-amylase and *α*-glucosidase by aqueous extract of morinda lucida benth leaf. *BioMed Research International*.

[12] Elya B., Basah K., Mun'Im A., Yuliastuti W., Bangun A., Septiana E. K. (2012). Screening of *α*-glucosidase inhibitory activity from some plants of Apocynaceae, Clusiaceae, Euphorbiaceae, and Rubiaceae. *Journal of Biomedicine and Biotechnology*.

[13] Shi Q.-W., Su X.-H., Kiyota H. (2008). Chemical and pharmacological research of the plants in genus *Euphorbia*. *Chemical Reviews*.

[14] Pintus F., Spano D., Mascia C., Macone A., Floris G., Medda R. (2013). Acetylcholinesterase inhibitory and antioxidant properties of *Euphorbia characias* latex. *Records of Natural Products*.

[15] Spanò D., Pintus F., Esposito F., Loche D., Floris G., Medda R. (2015). Euphorbia characias latex: micromorphology of rubber particles and rubber transferase activity. *Plant Physiology and Biochemistry*.

[16] Pintus F., Spano D., Corongiu S., Floris G., Medda R. (2011). Purification, primary structure, and properties of *Euphorbia characias* latex purple acid phosphatase. *Biochemistry*.

[17] Dainese E., Sabatucci A., Pintus F. (2014). Domain mobility as probed by small-angle X-ray scattering may account for substrate access to the active site of two copper-dependent amine oxidases. *Acta Crystallographica Section D: Biological Crystallography*.

[18] Spanò D., Pospiskova K., Safarik I. (2015). Chitinase III in *Euphorbia characias* latex: purification and characterization. *Protein Expression and Purification*.

[19] Pintus F., Medda R., Rinaldi A. C., Spanò D., Floris G. (2010). *Euphorbia* latex biochemistry: complex interactions in a complex environment. *Plant Biosystems*.

[20] Palomino-Schätzlein M., Escrig P. V., Boira H., Primo J., Pineda-Lucena A., Cabedo N. (2011). Evaluation of nonpolar metabolites in plant extracts by 13C NMR spectroscopy. *Journal of Agricultural and Food Chemistry*.

[21] Escrig P. V., Iglesias D. J., Corma A., Primo J., Primo-Millo E., Cabedo N. (2013). *Euphorbia characias* as bioenergy crop: a study of variations in energy value components according to phenology and water status. *Journal of Agricultural and Food Chemistry*.

[22] Pisano M. B., Cosentino S., Viale S. (2016). Biological activities of aerial parts extracts of *Euphorbia characias*. *BioMed Research International*.

[23] Pintus F., Spanò D., Corona A., Medda R. (2015). Antityrosinase activity of *Euphorbia characias* extracts. *PeerJ*.

[24] Prior R. L., Hoang H., Gu L. (2003). Assays for hydrophilic and lipophilic antioxidant capacity (oxygen radical absorbance capacity (ORACFL)) of plasma and other biological and food samples. *Journal of Agricultural and Food Chemistry*.

[25] Mosmann T. (1983). Rapid colorimetric assay for cellular growth and survival: application to proliferation and cytotoxicity assays. *Journal of Immunological Methods*.

[26] Huang H.-C., Hsieh W.-Y., Niu Y.-L., Chang T.-M. (2014). Inhibitory effects of adlay extract on melanin production and cellular oxygen stress in B16F10 melanoma cells. *International Journal of Molecular Sciences*.

[27] Horai H., Arita M., Kanaya S. (2010). MassBank: A public repository for sharing mass spectral data for life sciences. *Journal of Mass Spectrometry*.

[28] Stobiecki M. (2000). Application of mass spectrometry for identification and structural studies of flavonoid glycosides. *Phytochemistry*.

